The article "Relationship between Serum FGF21 and vWF Expression and Carotid Atherosclerosis in Elderly Patients with Hypertension" was published in 2022. Journal: J Healthc Eng.

# Relationship between Serum FGF21 and vWF Expression and Carotid Atherosclerosis in Elderly Patients with Hypertension

**DOI:** 10.1155/2022/6777771

**Published:** 2022-02-22

**Authors:** Jing Bian, Lairong Chen, Qin Li, Yunfeng Zhao, Delu Yin, Shanhong Sun

**Affiliations:** ^1^Department of Cardiovascular Medicine, the Affiliated Hospital of Kangda College of Nanjing Medical University (the First People's Hospital of Lianyungang), Lianyungang 222002, Jiangsu, China; ^2^Imaging Department, the Fourth People's Hospital of Lianyungang, Lianyungang 222002, Jiangsu, China

## Abstract

Cardiovascular (CV) and cerebrovascular (CBV) diseases are common in the elderly and cause severe damage, with high morbidity, disability, and mortality. Hypertension, as a risk factor for a variety of CV and CBV diseases, also affects many elderly patients. This study aimed to investigate the relationship between serum FGF21 and vWF expression and carotid atherosclerosis (CAS) in elderly patients with hypertension. We recruited 143 elderly hypertensive patients admitted to our hospital from July 2017 to November 2019 to this study, including 75 patients with comorbid CAS (the observation group, OG) and 68 patients without CAS (the control group, CG). Enzyme-linked immunosorbent assay (ELISA) was used to test serum expression levels of FGF21 and vWF; receiver operating characteristic (ROC) curves to evaluate the value of FGF21 and vWF in diagnosing CAS and predicting the 6-month prognosis in elderly hypertensive patients; Pearson's correlation analysis to analyze the correlation of FGF21/vWF with the plaque thickness and stenosis area in hypertensive patients with CAS. The incidence of CV and CBV events was markedly higher in the high FGF21/vWF group than in the low FGF21/vWF group. Patients from OG were divided into the high FGF21/vWF group and the low FGF21/vWF group based on the median expression level of FGF21/vWF, then the incidence of cardiovascular (CV) and cerebrovascular (CBV) events was compared between the high and low expression groups. Serum levels of FGF21 and vWF were markedly higher in patients from OG than in patients from CG. Both FGF21 and vWF were in positive correlation with the plaque thickness and stenosis area in patients from OG. The area under the ROC curve (AUC) for diagnosing CAS was 0.790 by FGF21 and 0.807 by vWF; the AUC for predicting the occurrence of CV and CBV events was 0.771 by FGF21 and 0.754 by vWF. Serum levels of FGF21 and vWF are increased in elderly patients with hypertension and comorbid CAS, so they can be used for diagnosing CAS and predicting prognosis.

## 1. Introduction

Cardiovascular (CV) and cerebrovascular (CBV) diseases are common in the elderly and cause severe damage, with high morbidity, disability, and mortality [1, 2]. Hypertension, as a risk factor for a variety of CV and CBV diseases, also affects many elderly patients [3]. Being hypertensive for a long time, patients have damaged vascular endothelial cells, altered tension in the walls of blood vessels, and accumulated monocytes, lymphocytes, and macrophages in the inner membrane, which decreases the elasticity of the arterial walls and makes them harder and thicker, so carotid atherosclerosis (CAS) is the most common complication among elderly patients with hypertension [4, 5].

The article "Relationship between Serum FGF21 and vWF Expression and Carotid Atherosclerosis in Elderly Patients with Hypertension" was published in 2022. Journal: J Healthc Eng.

A previous study reveals that patients with CAS are at high risk of CV diseases and emphasizes the importance of a timely diagnosis of CAS [6]. Abnormal platelet adhesion, severe vascular inflammation, and oxidative stress will participate in the formation of arterial thrombosis and atherosclerosis [7]. Atherosclerosis is a systemic diffuse pathological state that involves coronary arteries, carotid arteries, and other arteries and small blood vessels, further inducing coronary heart disease and stroke. Fibroblast growth factor 21 (FGF 21), an oxidative stress regulator that controls lipid and energy metabolism and serum metabolic parameters, can reduce hyperglycemia and dyslipidemia, mitigate CV diseases, and regulate oxidative stress [8, 9]. Von Willebrand factor (vWF) is a macromolecular protein-polymer released from damaged vascular endothelial cells into the blood circulation, which can induce platelet aggregation and adhesion, activate coagulation factors, and stimulate blood hypercoagulation, generally working as a marker of vascular endothelial injury [10, 11]. The study by Katneni and his team [12] suggests that vWF and its cleavage protease ADAMTS-13 play important roles during hemostasis and they also participate in the process of neonatal thrombosis. The relationship between serum FGF21 and vWF expression and CAS in elderly patients with hypertension remains unclear.

This study evaluated the diagnostic value of FGF21 and vWF for CAS in elderly hypertensive patients and analyzed their correlation with CAS.

## 2. Materials and Methods

### 2.1. Basic Information of Patients

We recruited 143 elderly hypertensive patients admitted to our hospital from July 2017 to November 2019 to this study, including 75 patients with comorbid CAS (the observation group, OG) and 68 patients without CAS (the control group, CG). OG was comprised of 53 males and 22 females at an average age of 51.6 ± 6.4 years, while CG was comprised of 44 males and 24 females at an average age of 52.3 ± 7.5 years. This study has obtained ethical approval from the Medical Ethics Committee of our hospital. All patients signed an informed consent form.

The article "Relationship between Serum FGF21 and vWF Expression and Carotid Atherosclerosis in Elderly Patients with Hypertension" was published in 2022. Journal: J Healthc Eng.

### 2.2. Inclusion and Exclusion Criteria

Inclusion criteria were as follows: patients diagnosed with hypertension according to the Guideline for the Prevention, Detection, Evaluation, and Management of High Blood Pressure in Adults proposed by the American Heart Association and American College of Cardiology in 2017 [13]; patients aged ≥60 years; patients with complete clinical data; and patients willing to cooperate with treatment and follow-up.

Exclusion criteria were as follows: patients attacked by CV and CBV events prior to admission, such as cerebral hemorrhage, cerebral infarction, sudden cardiac death, and acute myocardial infarction; patients with abnormal functions of the liver, kidney, and thyroid; and patients with coagulation dysfunction and immune dysfunction.

### 2.3. Detection Method

We collected 5 mL of venous blood from each patient in a sterilized environment at 7 am. The next morning, after admission, it was stored in the anticoagulation tube. The blood was immediately centrifuged at 3,000 xg at 4 °C for 10 minutes to collect the serum, and then the serum was stored at -80 °C. Serum expression levels of FGF21 and vWF were determined by enzyme-linked immunosorbent assay (ELISA), and the ELISA kits were purchased from Abcam (Cambridge, UK, item numbers: ab222506 and ab108918). Blank, standard, and sample wells were set, with 100 µl of sample diluent in each blank well, 100 µl of standard in each standard well, and 100 µl of sample in each sample well. The ELISA plate was sealed and incubated at 37 °C for 90 minutes. The liquid in each well was discarded, and then 100 *μ*l of biotin antibody working solution was added to each well, followed by incubation of the sealed ELISA plate at 37 °C for 1 hour. Subsequently, the liquid in each well was removed, and the plate was washed 3 times. The wells were dried, and 100 µl of enzyme conjugate was added to each well, followed by incubation at 37 °C for 30 minutes. Then, the liquid was removed, and the plate was washed five times. After that, 90 *μ*l of chromogenic reagent was added to each well, followed by incubation at 37 °C for 15 minutes in the dark. Finally, 50 *μ*l of stop solution was added to each well, and the optical density value of each well was determined at a wavelength of 450 nm within 15 minutes.

### 2.4. Follow-Up

Patients from OG were followed up for 6 months by telephone and follow-up visits. The CV and CBV events occurring during the follow-up period were recorded and filed every two months, including cerebral hemorrhage, cerebral infarction, sudden cardiac death, and acute myocardial infarction.

The article "Relationship between Serum FGF21 and vWF Expression and Carotid Atherosclerosis in Elderly Patients with Hypertension" was published in 2022. Journal: J Healthc Eng.

### 2.5. Outcome Measures

#### 2.5.1. Primary Outcome Measures

The primary outcome measures were as follows: the expression levels of FGF21 and vWF in the two groups of patients; the value of FGF21 and vWF for diagnosing CAS in elderly hypertensive patients with CAS; and predicting the 6-month prognosis according to the ROC curves.

#### 2.5.2. Secondary Outcome Measures

The secondary outcome measures were as follows: the correlation of FGF21 and vWF with the plaque thickness and stenosis area in patients from OG; the incidence of CV and CBV events in the high and low FGF21/vWF expression groups.

### 2.6. Statistical Analysis

All statistical calculations were performed on SPSS20.0 (SPSS Inc., Chicago, IL, USA). Count data was analyzed by the chi-square test, represented by x^2^. All the measurement data followed the normal distribution and was analyzed by the independent sample *t*-test. The correlation of FGF21 and vWF with the plaque thickness and stenosis area in patients from OG was tested by the Pearson correlation analysis. The value of FGF21 and vWF for diagnosing CAS in elderly hypertensive patients with CAS and predicting the 6-month prognosis was analyzed by the ROC curves. *P* < 0.05 indicates the difference is statistically significant.

## 3. Results

### 3.1. Baseline Data

The comparison of baseline data between OG and CG revealed no statistical differences in sex, age, BMI, diabetes, hyperlipidemia, smoking history, SBP, DBP, uric acid, and blood sugar, as shown in Table 1.

### 3.2. Expression Levels of FGF21 and vWF

Serum expression levels of FGF21 and vWF were markedly higher in OG than in CG (*P* < 0.05). The AUC for diagnosing CAS was 0.790 by FGF21, 0.807 by vWF, and 0.875 by the combined diagnosis, as shown in Figure 1 and Table 2.

### 3.3. Correlation of FGF21 and vWF with CAS

According to the Pearson correlation results, FGF21 levels were positively correlated with vWF levels in OG, and both FGF21 and vWF were in positive correlation with the plaque thickness and stenosis area in OG. More details are shown in Figure 2.

### 3.4. Incidence of CV and CBV Events

Patients from OG were divided into the high FGF21/vWF group and the low FGF21/vWF group based on the median expression level of FGF21/vWF. The incidence of CV and CBV events was markedly higher in the high FGF21/vWF group than in the low FGF21/vWF group, as shown in Table 3.

### 3.5. Prognostic Value of FGF21 and vWF

Patients in OG were divided into the excellent prognosis group and the poor prognosis group according to the presence of CV and CBV events. On the ROC curves, the AUC for predicting prognosis was 0.771 for FGF21 and 0.754 for vWF, as shown in Figure 3.

The article "Relationship between Serum FGF21 and vWF Expression and Carotid Atherosclerosis in Elderly Patients with Hypertension" was published in 2022. Journal: J Healthc Eng.

## 4. Discussion

Hypertension can cause pathological changes in multiple target organs such as the heart, brain, and kidneys. Furthermore, it leads to changed vascular physiology, damaged intima, remodeled vascular structure, hypertrophic vessel walls, and increased lipid content in the arterial wall, thereby causing plaques [14, 15]. A previous study reveals that patients with CAS are at high risk of CV diseases and emphasizes the importance of a timely diagnosis of CAS [6]. Atherosclerosis is a systemic diffuse pathological state that involves coronary arteries, carotid arteries, and other arteries and small blood vessels, further inducing coronary heart disease and stroke [16]. A former study suggests that immune response and inflammatory response are essential in the occurrence and development of atherosclerosis because some inflammatory mediators produced by macrophages aggravate inflammation of plaques, activate blood vessel walls to cause the instability of plaques, and induce thrombus [17].

In this study, serum levels of FGF21 and vWF were markedly higher in OG than in CG, indicating that FGF21 and vWF expression levels are increased significantly in hypertensive patients with CAS. As a biomarker of endothelial injury, vWF is highly expressed in patients with hypertension, diabetes, and other endothelial dysfunction diseases and poses a great impact on vascular permeability [18]. FGF21 is effective in relieving inflammation, reducing damage, and regulating glycolipids. Patients with CAS have markedly aggravated body damage and inflammation, which causes a compensatory increase in FGF21 levels. The study by Jin and his team [19] indicates that diabetic patients with arteriosclerosis, macrovascular, or microvascular undergo an increase in circulating FGF21 levels, especially in the early stage of atherosclerosis, and regards this increase as a compensatory upregulation, which is consistent with the results of this study. Based on the differences in FGF21 and vWF levels between the two groups, we speculated that FGF21 and vWF may have a certain diagnostic value for CAS in elderly hypertensive patients. Then, we plotted ROC curves and noted the favorable diagnostic value of FGF21 and vWF for CAS (an AUC of 0.790 by FGF21, 0.807 by vWF, and 0.875 by combined diagnosis), indicating that the combined diagnosis of FGF21 and vWF can achieve better diagnostic efficiency. A previous study reveals that the FGF21 levels are markedly enhanced in hypertensive patients and can be reduced by antihypertensive treatment [20].

Then, we analyzed the correlation between the expression levels of FGF21 and vWF in OG and their correlation with the plaque thickness and stenosis area. FGF21 levels were positively correlated with vWF levels in OG and both FGF21 and vWF were in positive correlation with the plaque thickness and stenosis area, suggesting that FGF21 and vWF levels increase as the severity of ACS increases. Hypertensive patients with comorbid CAS have a markedly higher risk of CV and CBV events [21]. We recorded the incidence of CV and CBV events in OG and found that the incidence of CV and CBV events was markedly higher in the high FGF21/vWF group than in the low FGF21/vWF group.

The article "Relationship between Serum FGF21 and vWF Expression and Carotid Atherosclerosis in Elderly Patients with Hypertension" was published in 2022. Journal: J Healthc Eng.

However, there are some problems in this study. For example, this study only recruited hypertensive patients and did not make a comparison between affected people and healthy people. Besides, this study did not investigate various targeted treatments for hypertension [22, 23], so the effects of these treatments on FGF21 and vWF levels are unclear. At present, the diagnosis of CAS is mainly achieved by imaging methods, such as carotid ultrasound [24, 25]. Here, we did not compare the differences between these diagnostic methods and FGF21 and vWF in diagnosing CAS. We will make such a comparison in the future and design a combined diagnosis by imaging methods and biomarkers to improve the diagnosis of CAS.

In summary, serum FGF21 and vWF levels are markedly higher in elderly hypertensive patients with CAS than in those without CAS, and the expression levels of FGF21 and vWF are in positive correlation with the severity of CAS.

## 5. Conclusion

However, there are some problems in this study. For example, we did not compare the differences between these diagnostic methods and FGF21 and vWF in diagnosing CAS. And also, this study only recruited hypertensive patients and did not make a comparison between affected people and healthy people. Besides, this study did not investigate various targeted treatments for hypertension [22, 23], so the effects of these treatments on FGF21 and vWF levels are unclear. At present, the diagnosis of CAS is mainly achieved by imaging methods, such as carotid ultrasound [24, 25]. We will make such a comparison in the future and design a combined diagnosis by imaging methods and biomarkers to improve the diagnosis of CAS.

In summary, serum FGF21 and vWF levels are markedly higher in elderly hypertensive patients with CAS than in those without CAS, and the expression levels of FGF21 and vWF are in positive correlation with the severity of CAS.

## Figures and Tables

**Figure 1:** Expression levels of FGF21 and vWF. (a) FGF21 levels are markedly higher in OG than in CG (*t* = 6.496, *p* < 0.001). (b) vWF levels are markedly higher in OG than in CG (*t* = 7.297, *p* < 0.001). ^*∗∗∗*^*P* < 0.001. (c) ROC curves demonstrate the diagnosis of CAS by FGF21 and vWF.

The article "Relationship between Serum FGF21 and vWF Expression and Carotid Atherosclerosis in Elderly Patients with Hypertension" was published in 2022. Journal: J Healthc Eng.

**Figure 2:** Correlation of FGF21 and vWF with CAS. (A) FGF21 is positively correlated with vWF (*r* = 0.793, *P* < 0.001). (B) FGF21 is positively correlated with the plaque thickness (*r* = 0.708, *P* < 0.001). (C) vWF is positively correlated with the plaque thickness (*r* = 0.780, *P* < 0.001). (D) FGF21 is positively correlated with the stenosis area (*r* = 0.741, *P* < 0.001). (E) vWF is positively correlated with the stenosis area (*r* = 0.744, *P* < 0.001).

**Figure 3:** Prognostic value of FGF21 and vWF. (a) On the ROC curve demonstrating the prediction of CV and CBV events in 6 months by FGF21, the AUC is 0.771, the sensitivity is 78.57%, and the specificity is 85.25%. (b) On the ROC curve demonstrating the prediction of CV and CBV events in 6 months by vWF, the AUC is 0.754, the sensitivity is 64.29%, and the specificity is 91.80%.

**Table 1:** Baseline data of the two groups.

		Observation group (*n* = 75)	Control group (*n* = 68)	t/*χ*^2^	P
Sex					
	Male	53 (70.67)	44 (64.71)	0.581	0.446
	Female	22 (29.33)	24 (35.29)		
Age (years)		51.6 ± 6.4	52.3 ± 7.5	0.602	0.548
BMI (kg/m^2^)		23.73 ± 1.82	24.2 ± 1.97	1.231	0.221
Diabetes					
	Yes	27 (36.00)	20 (29.41)	0.702	0.402
	No	48 (64.00)	48 (70.59%)		
Hyperlipidemia					
	Yes	17 (22.67)	12 (17.65)	0.556	0.456
	No	58 (77.33)	56 (82.35)		
Smoking history					
	Yes	28 (37.33)	21 (30.88)	0.659	0.417
	No	47 (62.67)	47 (69.12)		
SBP (mmHg)		168.87 ± 14.63	172.59 ± 17.25	1.395	0.165
DBP (mmHg)		113.47 ± 12.64	109.83 ± 11.49	1.795	0.075
Uric acid (*μ*mol/L)		252.93 ± 54.41	237.23 ± 46.62	1.844	0.067
Blood sugar (mmol/L)		6.47 ± 2.21	6.22 ± 1.96	0.713	0.477

*Note.* BMI: body mass index; SBP: systolic blood pressure; DBP: diastolic blood pressure.

**Table 2:** Parameters of ROC curves.

	AUC	95% CI	Sensitivity (%)	Specificity (%)	Youden index	Cut-off value
FGF21	0.790	0.714–0.866	76.00%	76.47%	52.47%	>428.82
vWF	0.807	0.737–0.877	62.67%	86.76%	49.43%	>149.76
Combined diagnosis	0.875	0.818–0.932	84.00%	80.88%	64.88%	>0.518

**Table 3:** CV and CBV events in the two groups.

	High FGF21 group (*n* = 38)	Low FGF21 group (*n* = 37)	X^2^	P
Cerebral hemorrhage	2 (5.26)	1 (2.70)		
Cerebral infarction	4 (10.53)	0 (0.00)		
Sudden cardiac death	1 (2.63)	0 (0.00)		
Acute myocardial infarction	5 (13.16)	1 (2.70)		
Overall incidence	12 (31.58)	2 (5.41)	8.459	0.004
Cerebral hemorrhage	High vWF group (*n* = 38)	Low vWF group (*n* = 37)		
	2 (5.26)	1 (2.70)		
Cerebral infarction	3 (7.89)	1 (2.70)		
Sudden cardiac death	1 (2.63)	0 (0.00)		
Acute myocardial infarction	5 (13.16)	1 (0.00)		
Overall incidence	11 (26.32)	3 (8.11)	5.362	0.021

The article "Relationship between Serum FGF21 and vWF Expression and Carotid Atherosclerosis in Elderly Patients with Hypertension" was published in 2022. Journal: J Healthc Eng.

## Data Availability

The datasets used and/or analyzed during the current study are available from the corresponding author on reasonable request.
